This article has been retracted.

# Principal Component and Path Analysis for Trait Selection Based on the Assessment of Diverse Lentil Populations Developed by Gamma-Irradiated Physical Mutation

**DOI:** 10.1155/2022/9679181

**Published:** 2022-07-18

**Authors:** Sandip Debnath, Abhik Sarkar, Kahkashan Perveen, Najat A. Bukhari, Kavindra Kumar Kesari, Amit Verma, Nihar Ranjan Chakraborty, Mulugeta Tesema

**Affiliations:** ^1^Department of Genetics and Plant Breeding, Institute of Agriculture, Visva-Bharati University, Sriniketan, PIN-731236 West Bengal, India; ^2^Department of Botany & Microbiology, College of Science, King Saud University, Riyadh 11495, Saudi Arabia; ^3^Department of Bioproducts and Biosystems, Aalto University, Espoo, P.O. Box 11000, Otakaari 1B, Finland; ^4^University Centre for Research & Development & Department of Computer Science & Engineering, Chandigarh University, Gharuan, Mohali, Punjab, India; ^5^Department of Chemistry (Analytical), College of Natural and Computational Sciences, DambiDollo University, Dambi Dollo, Oromia Region, Ethiopia

## Abstract

Lentil is a notable legume crop valued for its high protein, vitamin, mineral, and amino acid (lysine and tryptophan) content. This crop has a narrow genetic base due to the formation of gene pool barriers during interspecific hybridization within and across species. Mutagenesis may be seen as a novel and alternative breeding technique for the production of new diversity. For the identification of new alleles, the creation of mutants followed by selection in subsequent generations would be necessary. Induction of mutation in lentil cv. *Moitree* by gamma rays therefore produced high variation for the majority of quantitative measures examined. Henceforth, principal component analysis (PCA) and path coefficient analysis were conducted to identify and exclude redundant mutant genotypes with similar traits as the success of breeding is dependent on understanding the relationship between morpho-agronomic traits and seed yield. As shown by the findings of this research, the total quantity of pods per mutant plant should be given considerable priority. The identified mutant genotypes, such as lines 24, 43, 28, 33, and 10, may be used as parents in future breeding or released directly following trials.

## 1. Introduction

In India, lentils (*Lens culinaris* Medik) are an important pulse crop. It belongs to the *Fabaceae* family and contains 14 chromosomes (2*n* = 2*x*). [1]. It is an annual edible legume with pods and seeds shaped like lenses and purses [2]. This is the oldest known legume [3]. It's grains contain necessary amino acids like lysine and tryptophan [4]. Currently, pulses, their significance in food and nutrition security, and sustainable agriculture are receiving more worldwide attention than ever before. Legumes are included among high-protein plant foods. It is spectacular to note that protein-rich meals are advised to consume regularly by mesothelioma patients whose appetites may be affected by chemotherapy, and nutritious diets give energy and help preserve muscular mass. Mesothelioma patients generally eat too little protein and calories to promote healing, boost immunity, and fight tiredness. A healthy mesothelioma diet may reduce stress, maintain weight and energy, combat infection, and control treatment-related side effects. Improving the quality of the high-protein legume “lentil” employing novel crop improvement techniques might thus play a significant role. Systematized evaluation is required for the genetic and agronomic improvement of lentil. It will remain the major objective of all breeding initiatives. Frequent use of conventional breeding techniques has decreased genetic diversity, which is a primary need for crop improvement projects. To achieve the aim of increasing genetic variability, new breeding procedures, such as induced mutagenesis, are necessary. In addition to genetic diversity, induced mutagenesis allows for the improvement of a specific trait without affecting the genetic composition as a whole [5, 6]. The “daylength bottleneck” constrained the flow of lentil germplasm into the *Indo-Gangetic* plain due to its narrow genetic base, which is less sensitive to photoperiod and more sensitive to temperature than landraces from West Asia, despite the fact that South Asia is home to half of the world's lentil cultivation [7]. In addition, the tiny and fragile flowers reduced the success rate of artificial hybridization by 20–50% due to the problems of emasculation and pollination, which resulted in mutant plant damage. As a result, cross-pollination of lentils has become a time-consuming procedure [8]. In addition, *Lens* was known for the formation of cross ability barriers during interspecific hybridization within and across species [9]. The interspecific hybridization is a technique of intercrossing two different species which have the same genus. This technique is useful for exploiting useful genes from raw species to improve the cultivated species. Eventually, these events resulted in the narrow genetic foundation of lentils. Several researchers have already recognized this narrow genetic base as the fundamental constraint on lentil yield [10]. In addition, adaptive specificity and recurrent failures to use several unproductive wild germplasms contribute to the failure of lentil genetic advancement [11]. Given the aforementioned conditions, mutagenesis may be viewed as a unique and supplemental breeding approach. It is capable of producing variants that does not exist in the genetic background of the organism. Consequently, mutagenesis may be exploited to improve a multitude of desirable traits in a mutant plant species [12, 13]. The development of mutants followed by selection in the next generations would be essential for the discovery of novel alleles and might be released directly as varieties or prebreeding material in the near future if proved to be commercially viable and agronomically advantageous [14]. Nonetheless, crop yield in general is a complex process arising from the interplay of several genes with diverse environmental implications that impact a wide range of phenotypes [15]. Successful mutant plant selection during breeding requires knowledge of the link between morpho-agronomic parameters and seed yield [16]. A path coefficient analysis was conducted to determine the nature of the link between yield and other variables, as well as the direct and indirect effects of different factors on yield. PCA is a statistical technique used to identify and eliminate duplicate genotypes with similar characteristics [17]. It allows for the natural classification of genotypes and gives an accurate indication of genotypic differences. The primary benefit of PCA is that each genotype may be assigned to only one group [18]. In addition, this test is used to categorize a large number of variables into important components and assess their contribution to the total variance [19]. So, PCA was done to determine how the various attributes were connected and to identify the traits that cosegregated. This enabled for the identification of the characteristics so that the selected M_4_ mutants could be utilized for crop development. Having in mind the limitations on lentil yield and the importance of optimizing physical mutagen, a multiyear-induced mutagenesis field experiment was conducted from 2017 to 2021 to increase the genetic diversity and yielding potential of lentil cultivars.

## 2. Materials and Methods

Approximately 5000 healthy seeds of lentil (Cultivar: *Moitree*), were irradiated with 250 Gy of gamma rays because the GR_50_ value for *Moitree* (published elsewhere) was calculated to be 217.2 Gy. The irradiation was applied at the RNARC, BCKV, West Bengal, India, where gamma chamber (GC-6000) was utilized. Using the mutant plant-to-progeny method, in 2018-2019, seeds from the M_1_ generation were sown in the next generation to grow the M_2_ population in the field mentioned above. To investigate the mutagenic impact of the previously delivered gamma irradiation doses, individual mutant plants were picked across the field based on their chlorophyll content and a variety of morphological traits. After ten days of germination, the potential mutants were tagged and recorded correctly. In 2019–2020, 433 agro-morphologically superior mutants with high production potential were chosen and produced in the M_3_ generation using the bulk breeding technique to reap the benefits of natural selection. The M_4_ generation was made up of 62 types of economically superior mutant types that were obtained from 433 M_3_ populations in 2020–21.

These 62 lentil mutant types were grown at the institutional agricultural farm during winters of 2020-2021, using a RCBD design with three replications. Apparently healthy and competitive five mutant plants were randomly selected from each plot, and data were obtained on fourteen distinct traits defined by Satpathy and colleagues [20]. Dewey and Lu's path coefficient analysis was used to examine the direct and indirect impacts of a variety of independent factors on seed yield. [21]. Windostat version 9.2 was applied for statistical studies involving correlation, route analysis, and PCA. Following the formula presented by Allard (1960), different genetic parameters were determined [22].

## 3. Results

Recent research on the genetic diversity of 50 distinct lentil germplasms, as well as the identification of the best heritable attributes from our laboratory, was published [20]. Examining the direct and indirect impacts of numerous characteristics on seed yield, as well as analyzing the pattern of variation in characters, classifying the traits, and exploring novel mutants, was the objective of this research.

### 3.1. Principal Component Analysis

PCA was used to evaluate the diversity of 14 traits.  Table 1 illustrates, based on the variable factor loadings, that the eight PC aspects explained 78.21 percent of the total variance.

Each principal component analysis shows the central variability of all attributes. 14.11 percent of the total variation was explained by the first main component (PC1). The factors with the largest loading on PC1 were grain yield/mutant plant, days to fifty percent blooming, harvest index, and mutant plant height. 12.54 percent of the variation was explained by the second main component (PC2). The variables mutant plant height, days to fifty percent flowering, days to fifty percent pod maturity, seeds/mutant plant, biomass/mutant plant, and weight of 100 seeds showed high positive support, whereas the remaining variables revealed substantial negative involvement. The third main component (PC3) accounted for 11.30 percent of the variance. The remaining five PCs explained just 9.91, 8.88, 7.99, 7.33, and 6.11 percent of the variance, respectively. A scree plot depicted the proportion of variation attributable to eigenvalues and principal components for each graphed PC (Figure 1).

PC 1 had the largest variance with an eigenvalue of 1.97, whereas the variance of the remaining principal components gradually declined. After the fourth PC, the line begins to straighten out, with minor differences across PCs. It is obvious from the graph that PC1 had the highest variance compared to the other four PCs; therefore, it may be advantageous to select lines for characters with a positive impact under PC1. The PC score for each component contains both positive and negative values. These scores may be employed to develop precise selection indices whose strength is dictated by the variation explained by each basic component [23]. A high PC score for a certain genotype in a specific component suggests that the mutant's variables have high values. We acquired the PCA scores (Table 2) for 62 lentil mutant variants in the first three principal components and referred to them as axes *X* vector (PCA-1), *Y* vector (PCA-2), and *Z* vector (PCA-3).

The squared distance of each genotype from these three axes was also calculated there. These PCA scores for mutant lineages were graphed to create a three-dimensional scatter picture (Figure 2).

Examining these findings indicated eight distinct clusters by Tocher method (Figure 3). Four of these clusters were shown to be mono-genotypic. The distribution pattern of mutants in these clusters was discovered to be random, with no agro-morphological diversity serving as a reference. Mutants with a more phenotypic variability were clustered in both the same and distinct classes.

### 3.2. Genetic Variability of the Mutant Population

Studies of the coefficient of variation revealed that the phenotypic coefficient variation (PCV) values were greater than those of the genotypic coefficient variation (GCV) for the majority of the traits, indicating that the environment influences these traits to some extent during both the vegetative and reproductive stages (Table 3). Secondary branches (number) per plant had the largest phenotypic coefficient variation (PCV) and genotypic coefficient variation (GCV) according to the research (70.85 percent and 60.32 percent, respectively). Biomass/mutant plant (57.21 percent) was followed by number of major branches (36.69 percent), seeds/pod (36.17 percent), seeds/mutant plant (35.25 percent), and pods/mutant plant (33.44 percent). Characters with a high GCV include biomass/mutant plant (24.3 percent), pods/mutant plant (21.86 percent), seeds/pod (20 percent), and mutant plant height (21.0 percent). The high values of PCV above GCV for the aforementioned features imply strong environmental influences; hence, when establishing a breeding program using this material, additional attention should be placed on these traits. The secondary branches (number) exhibited the highest heritability and genetic advance as a percentage of the mean (72.47 percent and 105.79 percent, respectively), and the other traits in which high heritability and high genetic advance were observed were weight of 100 seeds, harvest index, and pods/mutant plant, indicating that these traits are less influenced by the environment and are more stable and governed by additive gene action. Consequently, the easy selection process affords these characters a larger potential for advancement.

### 3.3. Path Analysis

The correlation coefficients between genotypic and phenotypic characteristics for fourteen traits are provided in (Tables 4 and 5). Days for pod initiation and pods/mutant plant (0.221∗∗ and 0.404∗∗) and number of main branches (0.155∗), root length (0.149∗), seeds/pod (0.159∗), and harvest index (0.155∗) are significantly and positively linked with grain production per plant at both levels, respectively. Secondary branches (number) (0.43∗∗) and biomass/mutant plant (0.144∗) were shown to be substantially and adversely associated to grain production per plant. The phenotypic analysis indicated only a significant and positive connection between grain yield and pods/mutant plant (0.246∗∗), seeds/mutant plant (0.399∗∗), and biomass/mutant plant (0.306∗∗). The correlation study demonstrated the link between the features; hence, the relationship between the numerous lentil traits will establish their relative importance for yield enhancement.

Path analysis based on phenotypic correlations found that all variables had direct positive impacts on grain production per mutant plant, except for number of main and secondary branches, days for pod initiation, root length, and harvest index, which had direct negative effects. The number of main and secondary branches, pods per plant, and harvest index demonstrated favorable indirect impacts of mutant plant height on grain yield (Table 6). The number of main branches had favorable indirect impacts on the secondary branches (number), days to 50% blooming and pod initiation, pods per plant, root length, seeds per pod, and biomass/mutant plant. The secondary branches (number) had both direct and indirect negative impacts on mutant plant height, days to 50% blooming and pod maturity, root length, seeds per pod, and seed weight per 100 seeds. Days to 50% blooming have negative indirect impacts on grain production via solely mutant plant height, main branch number, and root length. The days to 50 percent blooming, the days for pod initiation, the weight of 100 seeds, and the harvest index are all negatively impacted by the days for pod initiation. Days for 50% pod maturity has a positive indirect influence on the number of main and secondary branches, days to 50% blooming and pod maturity, seeds per plant, and 100 seed weight. Pods per plant, on the other hand, have a negative indirect influence through just the number of main and secondary branches, days for pod initiation and 50% maturity, and seeds per pod. Through the secondary branches (number), pods per plant, root length, seeds per pod, biomass/mutant plant, and 100 seed weight, root length has a negative indirect effect. Seeds per pod have a positive indirect influence on secondary branch number, days to 50% blooming, root length, seeds per pod, seeds per plant, and biomass/mutant plant. Through mutant plant height, secondary branches (number), days for pod initiation, root length, and harvest index, seeds per plant have a negative indirect influence. Biomass/mutant plant has a negative indirect influence on mutant plant height, the number of main and secondary branches, the number of days before pod initiation, and pod maturity at 50 percent. There is a positive indirect impact of 100 seed weight on all variables except mutant plant height and seeds/pod. The harvest index has a favorable indirect impact via the secondary branches (number), days for 50% pod maturity, root length, seeds per pod, and seeds per plant.

Path analysis based on genotypic correlations revealed direct positive effects of mutant plant height, days to 50 percent pod maturity, pods/mutant plant, seeds/pod, biomass/mutant plant, and direct negative effects of primary branches (number), secondary branches (number), and days to 50 percent flowering, days for pod initiation, root length, seeds/mutant plant, 100 seed weight, and harvest index on grain yield (Table 7). The mutant plant height had favorable indirect impacts on grain production via the number of main branches, the secondary branches (number), the number of seeds per plant, the weight of 100 seeds, and the harvest index. Number of main branches had favorable indirect impacts via secondary branches (number), days for pod initiation, days for 50% pod maturity, pods per plant, root length, biomass/mutant plant, and 100 seed weight. The secondary branches (number) had negative direct and indirect impacts on mutant plant height, days to 50 percent pod maturity, root length, seeds per pod, and seeds per plant. Days to 50% blooming have indirect favorable benefits on grain output via mutant plant height, secondary branches (number), pods per plant, and root length. Days for pod initiation has a negative indirect influence on grain yield through days to 50% blooming, seeds per pod, seeds per plant, and harvest index. The secondary branches (number), the number of days to 50 percent blooming, the number of seeds per pod, and the number of seeds per plant have a positive indirect influence on the days to 50 percent pod maturity. In contrast, pods per plant have a beneficial indirect benefit through biomass/mutant plant and hundred seed weight. Root length has a negative indirect influence through the amount of secondary branches, seeds per pod, seeds per plant, and weight per 100 seeds. Seeds per pod have a negative indirect influence on three traits: mutant plant height, pods per plant, and harvest index. Through pods/mutant plant, seeds/pod, and biomass/mutant plant, seeds/mutant plant have a positive indirect impact. The days to 50% blooming, pods/mutant plant, seeds/pod, and harvest index indicate a favorable indirect influence of biomass/mutant plant. 100 seed weight demonstrates a beneficial indirect impact via the number of main and secondary branches, days for pod initiation and 50% pod maturity, biomass/mutant plant, and harvest index. The harvest index demonstrates a negative indirect influence via mutant plant height, number of main branches, days to 50% blooming and pod commencement, seeds/mutant plant, and biomass/mutant plant.

## 4. Discussion

It is suggested that PCA is useful for selecting agronomically superior mutant lines for breeding endeavors [24]. In multivariate analysis, PCA is the major selection method as well clustering using the Tocher technique separated the mutagenic populations in the current research, demonstrating that mutagenic treatments created diverse populations. Because analyzing several phenotypic traits is a time-consuming and error-prone procedure that might hamper selection; consequently, multivariate analysis is essential for accurate selection [25]. It also facilitates the reduction of complicated data and improves breeding accuracy. Within the various clusters, genetically distinct groups were categorized. In lentil improvement projects focused at promoting genetic variability, mutants selected from distinct clusters might thus be advanced to next generations [26]. Positive correlations were found between the first principal component and grain yield/mutant plant, days to fifty percent flowering, harvest index, mutant plant height, main branches (number), days for pod initiation, pods/mutant plant, and seeds/mutant plant, indicating that these variables fluctuate in the same direction. Therefore, the property of the high-yield mutant plant-1 is related to yield attribute traits and blooming traits. The PCA analysis demonstrated that yield contributed the most to population divergence, indicating that yield favorably responded to mutagenic treatments for the prospective selection of high-yield mutants. Similar modifications were applied to the second primary component, an evaluation of the architectural and floral aspects of mutant plants. The third key element emphasized the correlation between mutant plant morphology and its relationship. The first five PCs in our analysis explained 56.76 percent of the total variance. The pattern of distribution also suggested that the mutant group exhibited a high degree of quantitative trait variation [27]. The yield-related properties of the M_4_ populations were characterized using principal component analysis in order to explain their phenotypes and identify superior high-yield mutant plants for multiplication. The number of uncorrelated variables have decreased due to the linear adjustment of the original variables. Yield per mutant plant and harvest index are major contributions to genetic divergence; selecting these traits in the following generation might result in mutants with more distinctive yield characteristics [23, 24]. The three-dimensional scatter plot illustrates the second component with the first. Mutant-24, Mutant-43, and Mutant-28 have high values for the first component; thus, we presume that they also have high values for the characteristics that are closely related to it. Therefore, mutant plants from this diverse blend of mutant lines associated with certain traits may be used as breeding parents to generate better lentil varieties [17].

Surprisingly substantial environmental influence was observed for almost all traits, which is rare when genetic variability parameters are assessed on extant cultivars that are assumed to be acclimatized and adaptable in their optimal agro-climatic zones [37]. These results pointed to the genetic uniqueness of the newly created mutant types, which must be acclimatized by determining their ideal growth circumstances and particular agronomic practices. Yield is a polygenic trait with a complicated mode of inheritance, and direct selection for yield is seldom successful. Therefore, correlations between quantitative characteristics are influenced by the small cumulative effects of numerous genes governing trait expression. In fact, in mutant breeding initiatives, correlation analysis between character combinations is crucial for assessing the impact of yield characteristics on overall yield [28]. So, it is essential to prioritize indirect selection, concentrating on yield-altering traits. A thorough understanding of the relationship between yield and yield characteristics is effectively understood from path analysis. By splitting the correlation coefficient into direct and indirect effects, path analysis provides more comprehensive information on the interrelationships of complex traits; hence, it has been used to define the selection criteria for genetic improvement. The nature of the relationship between yield and its associated characteristics would decide which attribute will be used in indirect selection to increase lentil production. According to the scale supplied by Lenka and Mishra, the major direct influences on grain yield were seeds/mutant plant, followed by biomass/mutant plant and pods/mutant plant [29]. The major difference in correlation and path analysis may be attributable to the fact that correlation simply calculates mutual association without addressing causes, while path analysis detects causes and evaluates their relative significance. Therefore, correlation and path analysis must be investigated to determine the precise relationship between attributes. Similar patterns were seen in terms of days to fifty percent blossom [30], pods per mutant plant [31], branches per mutant plant [32], seeds per mutant plant [33], and biomass/mutant plant [34]. The disparity between direct impacts and genotypic correlations of traits revealed that the relationship was mostly the result of indirect effects of characteristics through other component variables. Therefore, indirect selection of the previously indicated feature is typically advantageous. By assigning correlations, previous research [35] differentiates between direct and indirect effects for a more exact evaluation of the cause-and-effect association. Several vegetative, yield, and yield-contributing factors have a high association, according to a recent study. These parameters have both direct and indirect impacts on pod yield and its contributing characteristics due to their interaction [36].

Therefore, it was discovered that mutation induction by gamma rays was useful for establishing new sources of variability in lentils and avoiding breeding limitations. The induction of mutation in cv. *Moitree* by 250 Gy of gamma rays resulted in considerable variance for the vast majority of quantitative parameters examined. Due to its significant connection with and direct impacts on seed yield per mutant plant, both PCA and path analysis suggested that selection should place a significant emphasis on the total number of pods per mutant plant. The findings of cluster analysis revealed that there are genetic differences among mutant families [37]. The found mutant genotypes, such as lines 24, 43, 28, 33, and 10, maybe employed as parents for future breeding.

## 5. Conclusion

Selecting superior crop genotypes requires genetic diversity. Artificial selection has reduced allelic diversity since time immemorial. So, extending genetic diversity in a crop species may improve breeding effectiveness. Mutagenesis may be introduced directly to elite cultivars without being disturbed by the circumstances of linkage drag. Therefore, a popular lentil cultivar was irradiated for this study. This approach uses irradiation to create diversity while retaining fertility. Consequently, this research helped to the discovery of significant variables that directly or indirectly affect lentil yields. The highlighted traits may serve as selection criteria for hybridization and continuous selection-based lentil yield enhancement programs. In addition, the researchers identified a number of lines with diverse sets of traits that may be used to create superior kinds. Induced mutations at loci controlling commercially relevant features in chosen high-yielding mutants have efficiently contributed to diversifying the existing lentil genetic base and will be of invaluable use for future lentil breeding programs. In the coming days, Targeting Induced Local Lesions in Genomes (TILLING) might be used to confirm the mutants generated by this study at the genomic level.

## Figures and Tables

**Figure 1:** Scree plot of eigenvalues and cumulative variability against different principal components in lentil mutants.

**Figure 2:** 3-D scatter diagram of PCA scores for mutant lines.

**Figure 3:** Distribution pattern of mutants in eight clusters by Tocher method.

**Table 1:** Eigenvalues for the first five principal components of various Lentil mutant characteristics.

	PC-1	PC-2	PC-3	PC-4	PC-5	PC-6	PC-7	PC-8
Eigenvalue	1.97542	1.75629	1.58303	1.3886	1.2444	1.11867	1.02712	0.85597
% variability explained	14.11013	12.5449	11.30738	9.91859	8.88858	7.99046	7.33658	6.11404
Cumulative variability explained	14.11013	26.65503	37.96241	47.881	56.76958	64.76005	72.09662	78.21066

Characters								
Mutant plant height (cm)	0.25048	0.38142	0.23943	0.35319	0.10706	0.23783	0.014	0.05966
Primary branches (number)	0.20003	-0.10371	-0.45645	0.03086	-0.04338	-0.27438	-0.45303	-0.28496
Secondary branches (number)	-0.42991	-0.36133	0.12583	0.21243	-0.12712	0.06455	-0.1351	-0.21038
Days for fifty percent flowering	0.33698	0.2377	-0.19927	-0.04982	-0.20773	-0.12079	-0.03962	-0.24344
Days for pod initiation	0.18892	-0.04746	0.05889	0.1501	-0.30677	0.08208	0.66552	-0.53522
Days for fifty percent pod maturity	-0.22596	0.21722	-0.18955	-0.00637	0.53665	-0.34055	0.12435	-0.43063
Pods/mutant plant	0.17953	-0.42745	-0.36813	0.02671	-0.3105	-0.13369	0.16883	0.26938
Root length (cm)	-0.20586	-0.03981	-0.32296	0.3199	0.24083	-0.27468	0.42932	0.28707
Seeds/pod	-0.09768	-0.29664	0.12013	-0.50335	0.28993	0.0991	0.20353	-0.01967
Seeds/mutant plant	0.05965	0.10157	0.36315	-0.22488	-0.21891	-0.64245	0.14612	0.23137
Biomass/mutant plant (g)	-0.28123	0.18136	-0.43314	-0.23535	-0.17822	0.42124	0.14436	0.06376
100 seed weight (g)	-0.22237	0.53104	-0.20035	-0.23379	-0.22218	-0.04262	0.06298	0.17617
Harvest index (%)	0.28529	-0.06901	-0.00689	-0.52825	0.13598	0.07246	0.05908	-0.13679
Grain yield/mutant plant (g)	0.46312	-0.07071	-0.15954	0.08975	0.39904	0.16212	0.1117	0.27769

**Table 2:** PCA scores of 62 lentil mutants shown as three axes *X* vector (PCA-1), *Y* vector (PCA-2), and *Z* vector (PCA-3).

	PCA I	PCA II	PCA III
Mutant types	*X vector*	*Y vector*	*Z vector*
1 | 1	-1.253	3.83	-4.81
2 | 2	-2.892	6.217	-4.34
3 | 3	0.173	5.999	-4.008
4 | 4	-0.26	7.368	-4.691
5 | 5	-0.077	8.372	-6.995
6 | 7	0.588	6.867	-5.029
7 | 13	-0.458	8.087	-5.493
8 | 14	-1.032	6.472	-5.597
9 | 23	-1.141	5.997	-5.395
10 | 25	0.223	6.772	-5.717
11 | 28	-1.393	6.023	-4.889
12 | 31	-0.641	6.329	-5.094
13 | 32	-1.49	9.11	-5.856
14 | 33	-0.31	7.795	-5.538
15 | 34	-1.247	7.855	-5.326
16 | 35	-1.05	7.798	-6.284
17 | 36	-1.013	7.083	-5.151
18 | 37	0.758	6.742	-5.443
19 | 38	1.296	6.264	-4.003
20 | 39	0.882	7.196	-5.277
21 | 40	0.117	8.701	-4.767
22 | 42	-0.12	6.11	-6.36
23 | 44	-0.401	6.081	-5.307
24 | 45	2.196	6.896	-4.829
25 | 47	-1.564	6.088	-4.856
26 | 51	-1.386	5.34	-4.572
27 | 52	-2.497	5.039	-5.712
28 | 59	1.275	6.306	-4.928
29 | 61	-1.038	5.948	-5.32
30 | 62	-1.195	5.985	-5.731
31 | 66	-1.172	4.713	-4.153
32 | 67	-1.217	7.502	-6.095
33 | 72	1.036	6.306	-5.251
34 | 76	0.057	5.592	-6.419
35 | 77	-1.16	5.831	-5.019
36 | 82	-0.029	7.121	-5.657
37 | 86	-0.982	6.165	-4.892
38 | 87	0.554	6.387	-6.6
39 | 88	-0.649	6.086	-5.168
40 | 89	-1.567	6.463	-5.268
41 | 91	0.326	4.788	-6.247
42 | 93	-0.109	5.682	-6.327
43 | 96	1.433	6.006	-5.533
44 | 97	0.44	6.565	-4.699
45 | 101	0.192	6.662	-5.335
46 | 103	-0.139	4.931	-3.679
47 | 104	-0.675	4.892	-5.731
48 | 105	-0.12	6.756	-6.362
49 | 107	0.069	6.586	-4.807
50 | 111	0.64	5.456	-5.767
51 | 114	-0.04	4.967	-5.511
52 | 115	-0.283	6.154	-6.45
53 | 116	0.934	4.987	-5.037
54 | 117	0.575	4.123	-5.015
55 | 127	-0.26	5.489	-5.362
56 | 128	-0.509	7.381	-5.841
57 | 133	0.819	5.802	-6.377
58 | 137	0.533	5.674	-5.441
59 | 138	-0.278	6.376	-5.838
60 | 142	0.35	6.519	-4.07
61 | 150	-0.303	6.729	-4.883
62 | 152	-0.761	6.008	-5.518

**Table 3:** Parameters related to genetic variability showing high influence of environment to most of the traits throughout both the vegetative and reproductive phases.

Genetic parameters	Mutant plant height (cm)	Main branches (number)	Secondary branches (number)	Days for 50% flowering	Days for pod initiation	Days for 50% pod maturity	Pods/mutant plant	Root length (cm)	Seeds/pod	Seeds/mutant plant	Biomass/mutant plant (g)	100 seed weight (g)	Harvest index (%)	Grain yield/mutant plant (g)
Heritability (%)	40.133	20.383	72.475	16.04	26.397	40.155	42.762	17.61	33.344	24.311	18.042	71.391	56.285	20.459
Genotypic coefficient of variations (GCV)	20.046	16.569	60.323	5.637	2.503	2.76	21.868	12.584	20.887	17.382	24.301	21.431	10.958	19.507
Phenotypic coefficient of variations (PCV)	31.642	36.699	70.858	14.075	4.872	4.355	33.441	29.988	36.171	35.253	57.21	25.364	14.607	43.127
Genetic advance	3.607	0.217	2.067	2.362	1.846	3.092	1.354	0.511	0.367	1.036	0.03	0.333	6.321	0.009
Genetic advance as % means	26.16	15.409	105.79	4.651	2.649	3.602	29.458	10.879	24.845	17.655	21.263	37.301	16.936	18.176

**Table 4:** Genotypic correlation coefficients between all investigated traits over 62 novel mutant types.

Traits	Mutant plant height (cm)	Main branches (number)	Secondary branches (number)	Days for 50% flowering	Days for pod initiation	Days for 50% pod maturity	Pods/mutant plant	Root length (cm)	Seeds/pod	Seeds/mutant plant	Biomass/mutant plant (g)	100 seed weight (g)	Harvest index (%)
Mutant plant height (cm)													
Main branches (number)	-0.392∗∗												
Secondary branches (number)	-0.213∗∗	-0.118^NS^											
Days for 50% flowering	0.162∗	0.360∗∗	-0.242∗∗										
Days for pod initiation	0.193∗∗	-0.196∗∗	-0.253∗∗	0.128^NS^									
Days for 50% pod maturity	-0.035^NS^	0.055^NS^	-0.222∗∗	-0.078^NS^	0.033^NS^								
Pods/mutant plant	-0.247∗∗	0.504∗∗	0.007^NS^	0.266∗∗	0.195∗∗	-0.383∗∗							
Root length (cm)	0.080^NS^	-0.144∗	0.172∗	-0.021^NS^	-0.081^NS^	0.508∗∗	0.244∗∗						
Seeds/pod	-0.213∗∗	-0.329∗∗	-0.069^NS^	-0.078^NS^	-0.053^NS^	0.111^NS^	-0.321∗∗	-0.346∗∗					
Seeds/mutant plant	-0.375∗∗	0.030^NS^	0.141^NS^	0.003^NS^	0.157∗	-0.178∗	0.441∗∗	0.153∗	0.107^NS^				
Biomass/mutant plant (g)	-0.497∗∗	0.107^NS^	0.108^NS^	-0.030^NS^	0.130^NS^	-0.287∗∗	0.285∗∗	0.128^NS^	0.259∗∗	0.114^NS^			
100 seed weight (g)	-0.052^NS^	-0.104^NS^	-0.136^NS^	0.221∗∗	-0.139^NS^	0.164∗	-0.108^NS^	0.081^NS^	-0.095^NS^	0.065^NS^	0.667∗∗		
Harvest index (%)	-0.080^NS^	0.126^NS^	-0.294∗∗	0.100^NS^	0.101^NS^	0.139^NS^	0.036^NS^	-0.291∗∗	0.378∗∗	0.113^NS^	-0.043^NS^	-0.218∗∗	
Grain yield/plant (g)	0.102^NS^	0.155∗	-0.430∗∗	0.049^NS^	0.221∗∗	-0.052^NS^	0.404∗∗	0.149∗	0.159∗	0.075^NS^	-0.144∗	0.005^NS^	0.155∗

∗ = significant at 5 percent level; ∗∗ =significant at 1 percent level; NS = Non-Significant.

**Table 5:** Phenotypic correlation coefficients between all investigated traits over 62 novel mutant types.

Traits	Mutant plant height (cm)	Main branches (number)	Secondary branches (number)	Days for 50% flowering	Days for pod initiation	Days for 50% pod maturity	Pods/mutant plant	Root length (cm)	Seeds/pod	Seeds/mutant plant	Biomass/mutant plant (g)	100 seed weight (g)	Harvest index (%)
Mutant plant height (cm)													
Main branches (number)	-0.179∗												
Secondary branches (number)	-0.051^NS^	-0.006^NS^											
Days for 50% flowering	-0.005^NS^	0.016^NS^	-0.065^NS^										
Days for pod initiation	0.067^NS^	-0.076^NS^	-0.147∗	-0.079^NS^									
Days for 50% pod maturity	-0.019^NS^	-0.121^NS^	-0.159∗	0.028^NS^	0.094^NS^								
Pods/mutant plant	0.031^NS^	0.108^NS^	0.026^NS^	0.127^NS^	0.037^NS^	-0.100^NS^							
Root length (cm)	0.018^NS^	-0.059^NS^	0.060^NS^	0.105^NS^	-0.003^NS^	0.111^NS^	-0.002^NS^						
Seeds/pod	-0.087^NS^	0.011^NS^	-0.053^NS^	0.014^NS^	0.060^NS^	-0.024^NS^	-0.292∗∗	-0.083^NS^					
Seeds/mutant plant	-0.069^NS^	-0.025^NS^	0.115^NS^	0.047^NS^	0.045^NS^	0.009^NS^	0.389∗∗	0.078^NS^	0.052^NS^				
Biomass/mutant plant (g)	-0.010^NS^	0.012^NS^	0.101^NS^	0.040^NS^	0.030^NS^	-0.059^NS^	0.297∗∗	-0.125^NS^	0.153∗	0.462∗∗			
100 seed weight (g)	-0.045^NS^	-0.077^NS^	-0.080^NS^	0.089^NS^	-0.062^NS^	0.077^NS^	0.016^NS^	-0.055^NS^	-0.048^NS^	0.111^NS^	0.336∗∗		
Harvest index (%)	-0.092^NS^	0.058^NS^	-0.206∗∗	-0.027^NS^	0.118^NS^	0.190∗∗	-0.008^NS^	-0.132^NS^	0.164∗	0.039^NS^	-0.114^NS^	-0.166∗	
Grain yield/plant (g)	0.073^NS^	-0.046^NS^	-0.101^NS^	0.045^NS^	0.053^NS^	0.046^NS^	0.246∗∗	-0.036^NS^	0.049^NS^	0.399∗∗	0.306∗∗	0.111^NS^	0.023^NS^

∗ = significant at 5 percent level; ∗∗ =significant at 1 percent level; NS = Non-Significant.

**Table 6:** Phenotypic path matrix based on phenotypic correlations for all the variables to reveal direct as well as indirect impacts on grain yield per mutant plant.

Phenotypic path matrix	Mutant plant height (cm)	Main branches (number)	Secondary branches (number)	Days for 50% flowering	Days for pod initiation	Days for 50% pod maturity	Pods/mutant plant	Root length (cm)	Seeds/pod	Seeds/mutant plant	Biomass/mutant plant (g)	100 seed weight (g)	Harvest index (%)	Grain yield/plant (g) *correlations*
Mutant plant height (cm)	0.40412	0.17438	0.06296	-0.02478	-0.05976	-0.02712	-0.34366	-0.05008	-0.05916	0.01869	-0.01555	0.00212	0.01956	*0.102^NS^*
Main branches (number)	-0.15849	-0.44463	0.03484	-0.05519	0.06077	0.04291	0.7006	0.0905	-0.09137	-0.00148	0.00336	0.00428	-0.03089	*0.155*∗
Secondary branches (number)	-0.08597	0.05234	-0.29594	0.03709	0.07828	-0.17306	0.00956	-0.10776	-0.01903	-0.00703	0.00339	0.00563	0.07209	*-0.430*∗∗
Days for 50% flowering	0.06541	-0.16024	0.07168	-0.15313	-0.03973	-0.061	0.36962	0.01306	-0.02156	-0.00015	-0.00095	-0.00913	-0.02456	*0.049^NS^*
Days for pod initiation	0.07805	0.08734	0.07488	-0.01967	-0.3094	0.02587	0.27033	0.05086	-0.01482	-0.0078	0.00406	0.00572	-0.02481	*0.221*∗∗
Days for 50% pod maturity	-0.01405	-0.02446	0.06565	0.01198	-0.01026	0.78004	-0.53172	-0.31886	0.03084	0.00888	-0.00898	-0.00674	-0.03401	*-0.052^NS^*
Pods/mutant plant	-0.09994	-0.22417	-0.00204	-0.04073	-0.06019	-0.29847	1.38963	-0.15324	-0.08911	-0.02197	0.00891	0.00445	-0.0089	*0.404*∗∗
Root length (cm)	0.03222	0.06406	-0.05077	0.00318	0.02505	0.39598	0.33903	-0.62812	-0.09612	-0.00763	0.004	-0.00335	0.07146	*0.149*∗
Seeds/pod	-0.08607	0.14627	0.02028	0.01188	0.01651	0.08662	-0.44584	0.21737	0.27776	-0.00532	0.0081	0.00393	-0.09285	*0.159*∗
Seeds/mutant plant	-0.15162	-0.01318	-0.04179	-0.00045	-0.04844	-0.13908	0.61281	-0.09618	0.02966	-0.04982	0.00356	-0.00269	-0.02779	*0.075^NS^*
Biomass/mutant plant (g)	-0.20088	-0.04774	-0.03208	0.00463	-0.0402	-0.22381	0.3956	-0.08034	0.07194	-0.00567	0.03128	-0.02748	0.01066	*-0.144*∗
100 seed weight (g)	-0.02082	0.04617	0.04039	-0.0339	0.04291	0.12755	-0.14996	-0.05098	-0.02651	-0.00325	0.02086	-0.04122	0.05343	*0.005^NS^*
Harvest index (%)	-0.03222	-0.05598	0.08695	-0.01533	-0.03129	0.10811	0.05038	0.18296	0.10511	-0.00564	-0.00136	0.00898	-0.24535	*0.155*∗

∗ = significant at 5 percent level; ∗∗ =significant at 1 percent level; NS = Non-Significant.

**Table 7:** Genotypic path matrix based on genotypic correlations for all the variables to reveal direct as well as indirect impacts on grain yield per mutant plant.

Genotypic path matrix	Mutant plant height (cm)	Main branches (number)	Secondary branches (number)	Days for 50% flowering	Days for pod initiation	Days for 50% pod maturity	Pods/mutant plant	Root length (cm)	Seeds/pod	Seeds/mutant plant	Biomass/mutant plant (g)	100 seed weight (g)	Harvest index (%)	Grain yield/plant (g) *correlations*
Mutant plant height (cm)	0.08526	0.00585	0.007	-0.00002	-0.00012	-0.00081	0.00329	-0.00076	-0.00389	-0.02223	-0.00122	-0.00073	0.00107	*0.073^NS^*
Main branches (number)	-0.0153	-0.03263	0.00077	0.00007	0.00014	-0.00527	0.01129	0.00251	0.00051	-0.00809	0.00149	-0.00125	-0.00068	*-0.046^NS^*
Secondary branches (number)	-0.00431	0.00018	-0.13852	-0.00027	0.00027	-0.00689	0.00276	-0.00257	-0.00237	0.03698	0.01274	-0.0013	0.00239	*-0.101^NS^*
Days for 50% flowering	-0.00047	-0.00053	0.00901	0.0042	0.00014	0.00122	0.01333	-0.0045	0.00061	0.01513	0.005	0.00145	0.00032	*0.045^NS^*
Days for pod initiation	0.00574	0.00249	0.02042	-0.00033	-0.0018	0.00409	0.00384	0.00013	0.00269	0.01441	0.00379	-0.00101	-0.00138	*0.053^NS^*
Days for 50% pod maturity	-0.0016	0.00396	0.02196	0.00012	-0.00017	0.04347	-0.01051	-0.00475	-0.00108	0.00287	-0.00741	0.00125	-0.00221	*0.046^NS^*
Pods/mutant plant	0.00267	-0.00351	-0.00364	0.00053	-0.00007	-0.00435	0.10493	0.00009	-0.01306	0.12471	0.03723	0.00025	0.00009	*0.246*∗∗
Root length (cm)	0.00151	0.00191	-0.0083	0.00044	0.00001	0.00481	-0.00022	-0.04292	-0.00372	0.02511	-0.01568	-0.00089	0.00153	*-0.036^NS^*
Seeds/pod	-0.00741	-0.00037	0.00733	0.00006	-0.00011	-0.00104	-0.03061	0.00357	0.04476	0.01676	0.01923	-0.00077	-0.00191	*0.049^NS^*
Seeds/mutant plant	-0.00591	0.00082	-0.01598	0.0002	-0.00008	0.00039	0.04083	-0.00336	0.00234	0.32051	0.05799	0.0018	-0.00045	*0.399*∗∗
Biomass/mutant plant (g)	-0.00083	-0.00039	-0.01405	0.00017	-0.00005	-0.00257	0.03112	0.00536	0.00686	0.14807	0.12553	0.00546	0.00132	*0.306*∗∗
100 seed weight (g)	-0.00383	0.00252	0.01111	0.00038	0.00011	0.00336	0.00165	0.00237	-0.00214	0.03552	0.04222	0.01622	0.00194	*0.111^NS^*
Harvest index (%)	-0.00783	-0.00189	0.02847	-0.00011	-0.00021	0.00826	-0.00081	0.00565	0.00733	0.01236	-0.01426	-0.0027	-0.01165	*0.023^NS^*

∗ = significant at 5 percent level; ∗∗ =significant at 1 percent level; NS = Non-Significant.

## Data Availability

The data shall be made available on request to the corresponding authors.
